# Deep Learning Reconstruction Algorithm-Based MRI Image Evaluation of Edaravone in the Treatment of Lower Limb Ischemia-Reperfusion Injury

**DOI:** 10.1155/2022/1408156

**Published:** 2022-08-31

**Authors:** Jianping Liu, Xunhong Duan, Rong Ye, Junqi Xiao, Cuifu Fang, Fengen Liu

**Affiliations:** ^1^Department of Vascular Surgery, First Affiliated Hospital of Gannan Medical College, Ganzhou 341000, Jiangxi, China; ^2^Key Laboratory of Prevention and Treatment of Cardiovascular and Cerebrovascular Diseases, Ministry of Education, Gannan Medical University, Ganzhou 341000, China

## Abstract

This research aimed to evaluate the therapeutic effect of edaravone on lower limb ischemia-reperfusion injury by MRI images of graph patch-based directional curvelet transform (GPBDCT), compression reconstruction algorithm. 200 patients with lower limb ischemia-reperfusion injury after replantation of severed limb were randomly divided into the observation group (edaravone treatment) and control group (Mailuoning injection treatment), with 100 cases in each group. MRI scanning and image processing using the GPBDCT algorithm were used to evaluate the therapeutic effect of the two groups of patients. The results showed that the signal noise ratio (SNR) (22.01), relative *l*_2_ norm error (RLNE) (0.0792), and matching degree *γ* (0.9997) of the compression and reconstruction algorithm based on GPBDCT were superior to those of the conventional compression and reconstruction algorithm (*P* < 0.05). MRI examination showed that the decrease of bleeding signal after treatment in the observation group was superior to that in the control group. The levels of superoxide dismutase (SOD) (15 ± 2.02), malondialdehyde (MDA) (2.27 ± 1.02), B cell lymphoma-2 (Bcl-2) (8.5 ± 1.02), Bcl-2-associated *X* (Bax) (3.7 ± 0.42), and Caspase-3 protein (35.9 ± 5.42) in the observation group before and after treatment were significantly higher than those in the control group (*P* < 0.05). In conclusion, the GPBDCT-based compression reconstruction algorithm has a better effect on MRI image processing, and edaravone can better remove free radicals and alleviate apoptosis.

## 1. Introduction

Limb ischemia-reperfusion injury refers to the pathological process of the damage of human limbs and the occurrence of ischemia-reperfusion, which leads to the further aggravation or even irreversible damage of the original symptoms such as abnormal metabolism, destruction of tissue structure, and dysfunction of the limbs [1]. It is commonly seen in the diseases such as limb replantation, osteofascial compartment syndrome, and vascular injury lesions of the limbs. Studies have shown that limb ischemia in the perfusion damage can cause oxygen free radical content increase, calcium overload, neutrophil increase, cell damage, and other manifestations, and free radical scavengers can reduce ischemia-reperfusion injury through a variety of ways [2–4]. Edaravone is a free radical scavenger, which is first used in the treatment of cerebral ischemia-reperfusion injury. The long-term clinical practice has proved that edaravone has a significant effect on the treatment of ischemic reperfusion injury [5, 6]. Mailuoning, as a traditional Chinese medicine preparation with antithrombotic and blood viscosity reduction, has a protective effect on limb ischemia-reperfusion injury, but there is a lack of research on the therapeutic effect between it and edaravone. In the examination methods of diseases, MRI has been increasingly applied in clinical imaging research with its advantages of noninvasiveness and high resolution. Moreover, with the rapid development of modern science and technology, it further promotes the application of MRI technology in ischemic reperfusion injury diseases [7]. However, there are few studies on the application of MRI in limb ischemia-reperfusion injury, most of them are about brain ischemia-reperfusion injury, and studies have shown that MRI can be well applied in the examination and diagnosis of such diseases.

In order to make the imaging technology more accurate in the diagnosis of diseases, imaging is often combined with deep learning algorithms in clinical examination [8, 9]. For MRI technology, some researchers have proposed a compressed sensing (CS) algorithm to reduce the amount of data sampling and save data storage space and computational time. Then, some experts introduced the CS algorithm into MRI technology to remove artifacts in the imaging, so as to improve MRI image clarity [10, 11]. However, the traditional CS reconstruction algorithm has limitations in image processing, which cannot completely suppress image noise and preserve image edge information. Therefore, some experts proposed the MRI image CS image reconstruction algorithm based on the curvelet transform of the image block to suppress the noise of the MRI image and retain the edge information [12], which achieved good application results. The above algorithm was used in this experiment.

200 patients with lower limb ischemia-reperfusion injury after limb amputation were selected as the research objects. The MRI examination images optimized by the compressive sensing image reconstruction algorithm based on image block curvelet transform were used as the evaluation means to evaluate the therapeutic effect of edaravone in the treatment of lower limb ischemia-reperfusion injury. It was to provide more effective treatment and reasonable research basis for patients with upper and lower limb ischemia-reperfusion injury.

## 2. Methods

### 2.1. Research Objects

200 patients with lower limb ischemia-reperfusion injury after limb replantation in hospital from September 2018 to September 2020 were selected, including 135 male patients and 65 female patients, with an age range of 22∼55 years and an average age of (37.45 ± 6.01) years. 200 patients were randomly divided into two groups, 100 cases in each group. A group of patients treated with edaravone was set as the observation group. The other group was treated with Mailuoning injection as the control group. This study was approved by the ethics committee of the hospital.

Inclusion criteria were as follows: patients who met the criteria for limb replantation and the time from injury to operation was less than 8 hours for all patients.

Exclusion criteria were as follows: patients with coagulation disorder and active bleeding; patients with organic lesions of the heart, liver, kidney, and other important organs; patients in special periods such as pregnancy, puerperium, or lactation; patients with a history of drug allergy such as edaravone and Mailuoning injection; patients with head, chest, and abdomen organ injury; limb soft tissue >1/4 of patients with limb cross-section; patients with open compound injury with vascular injury; patients with thrombosis-obstructive vascular disease of limbs or primary deep venous valve disease; and patients with mental disorders.

### 2.2. MRI Examination

3.0T magnetic resonance equipment was used. First, patients were guided to relax, and then, a scan was performed. Before scanning, the patients performed a plain scan to determine the disease location, and the coronal scan was performed. The scanning sequences included T1-weighted imaging (T1WI), T2-weighted imaging (T2WI), and dynamic contrast enhanced-MRI (DEC-MRI). Specific scan sequence parameters are shown in Table 1.

### 2.3. CS Image Reconstruction Algorithm Based on Curvelet Transform of Image Block

#### 2.3.1. CS and MRI

The CS reconstruction algorithm of MRI images essentially solves the problem of *l*_1_ norm optimization, as shown in the following equation.

(1) $$\begin{array}{c} \underset{\partial }{\text{min}}{\left\|\partial \right\|}_{1}s.t.y=℘F_{U\partial }. \end{array}$$

In the above equation, ‖*∂*‖_1_ in the *l*_1_ norm is the sum of absolute values of all elements in the vector *∂*. *℘* is the sparse transform coefficient, and *F*_*U*_ is the initial MRI image. When the alternating direction optimization algorithm is widely used in MRI image reconstruction, the optimization problem in (1) is transformed.

(2) $$\begin{array}{c} \underset{\alpha }{\text{min}\frac{1}{2}}\left\|y-F_{U\alpha 2}^{2}\right\|+\beta {\left\|\emptyset^{H}\alpha \right\|}_{1}, \end{array}$$

where ∅^*H*^ is the sparse transformation, *F*_*Uα*_ is the reconstructed MRI images; *β* is the sparse coefficient of MRI image, and *y* is the obtained *k* spatial data.

#### 2.3.2. CS Image Reconstruction Based on Directional Curvelet Transform of Image Block

The first is the application of graph patch-based directional curvelet transform (GPBDCT). Under GPBDCT, the results of the MRI image block are shown in Figure 1.

It is supposed that *φ*^*T*^ is the two-dimensional forward curvelet transform of the image *X*, and *Q*_*i*_ is the transform coefficient *φ*^*T*^*X* of the image. *X* is divided into blocks, *ai*=*Q*_*i*_*φ*^*T*^*X*(1,2,…, *I*). In addition, the candidate's direction set *x*={*x*_1_, *x*_2_,…, *x*_*c*_,…, *x*_*C*_}.

(3) $$\begin{array}{c} \zeta_{i,c}=\underset{x_{i,c}\in x}{\text{arg min}}{\left\|{\bar{b}}_{i,c}\left(x_{i,c},E\right)-\emptyset^{T}P\left(x_{i,c}\right)Q_{i}\varphi^{T}X\right\|}_{2}^{2}, \end{array}$$

where ∅^*T*^ is the positive transform of one-dimensional orthogonal Radon transform, *i* is the number of blocks of MRI images, *E* is the number of curvature coefficients, ${\bar{b}}_{i,c}\left(x_{i,c},E\right)$ is the largest *E* coefficients of the curvature coefficients ∅^*T*^*P*(*x*_*i*,*c*_)*Q*_*i*_*φ*^*T*^*X*, *x*_*i*,*c*_ is the *c* candidate direction of the *i* block, and *P*(*x*_*i*,*c*_) is the direction *x*_*i*,*c*_ parallel rearranged pixels. The coefficients *z* in the directional curvelet transform domain of image block in the image *X* are as follows.

(4) $$\begin{array}{c} z=\left[\partial_{1},\ldots ,\partial_{i},\ldots ,\partial_{I}\right],\\ z=\left[\emptyset^{T}P\left(\xi_{1}\right)Q_{1},\ldots ,\emptyset^{T}P\left(\xi_{i}\right)Q_{i},\ldots ,\emptyset^{T}P\left(\xi_{I}\right)Q_{I}\right]\varphi^{T}X,\;\\ \varphi^{T}X=B_{ℑ}X,\\ X=\frac{1}{p}B_{ℑ}^{T}X, \end{array}$$

where *p* is the overlap coefficient of each pixel.

PBDCT is imported into the CS reconstruction algorithm, and the norm *l*_0_ is used to achieve image reconstruction with less measured values. The specific expressions are as follows.

(5) $$\begin{array}{c} \bar{\bar{X}}=\text{arg min}{\left\|B_{ℑ}X\right\|}_{0}+\frac{\beta }{2}{\left\|y-F_{U}X\right\|}_{2}^{2}. \end{array}$$

Among them, *F*_*U*_ is the Fourier undersampling operator, *y* is the spatial sampling data, ‖*B*_*ℑ*_*X*‖_0_ is the image binding items, ‖*y* − *F*_*U*_*X*‖_2_^2^ is the data validation items, and *β* is the weight of balancing ‖*B*_*ℑ*_*X*‖_0_ and ‖*y* − *F*_*U*_*X*‖_2_^2^.

In order to make the calculation process easier, the auxiliary variable *∂*_*i*_=∅^*T*^*P*(*ξ*_*i*_)*Q*_*i*_*X* is subjected into (5).

(6) $$\begin{array}{c} \underset{X,\partial_{i}}{\text{min}}\sum_{i=1}^{I}\left({\left\|\partial_{i}\right\|}_{1}+\frac{\eta }{2}{\left\|\partial_{i}-\emptyset^{T}P\left(\xi_{i}\right)Q_{i}X\right\|}_{2}^{2}+\frac{1}{2}{\left\|y-F_{U}X\right\|}_{2}^{2}\right). \end{array}$$

According to (6), if *η* increased, the solution of the previous *η* value is the initial solution of the next  *η*. If the *η* value is certain, the solving process is as follows.

The first step: determining the *X* value and solving each *∂*_*i*_ value,

(7) $$\begin{array}{c} \underset{X,\partial_{i}}{\text{min}}{\left\|\partial_{i}\right\|}_{1}+\frac{\eta }{2}{\left\|\partial_{i}-\emptyset^{T}P\left(\xi_{i}\right)Q_{i}X\right\|}_{2}^{2}. \end{array}$$

In (7), *∂*_*i*_ is calculated by soft threshold.

(8) $$\begin{array}{c} \bar{\partial_{i}}=E\left({\left(Q_{i}P\left(\bar{x_{i}}\right)\emptyset \right)}^{T}X,\frac{1}{\mu }\right). \end{array}$$

Step 2: determining all *∂*_*i*_ values,

(9) $$\begin{array}{c} \underset{X}{\text{min}}\sum_{i=1}^{I}\left(\frac{\eta }{2}{\left\|\partial_{i}-\emptyset^{T}P\left(\xi_{i}\right)Q_{i}X\right\|}_{2}^{2}\right)+\frac{1}{2}{\left\|y-F_{U}X\right\|}_{2}^{2}. \end{array}$$

The above equation is solved by the regularization equation.

(10) $$\begin{array}{c} \left(\eta \sum_{i=1}^{I}Q_{i}^{T}P^{T}\left(\bar{x_{i}}\right)\emptyset \emptyset^{T}P\left(\xi_{i}\right)Q_{i}+\beta F_{U}^{H}F_{U}\right)X=\eta \sum_{i=1}^{I}Q_{i}^{T}P^{T}\left(\bar{x_{i}}\right)\emptyset \partial_{i}+\beta F_{U}^{H}y\left(\frac{\eta }{2}{\left\|\partial_{i}-\emptyset^{T}P\left(\xi_{i}\right)Q_{i}X\right\|}_{2}^{2}\right), \end{array}$$

where ∅∅^*T*^=*L*,$P^{T}\left(\bar{x_{i}}\right)P\left(\bar{x_{i}}\right)=L$. Equation (10) can also be simplified as follows.

(11) $$\begin{array}{c} \eta \sum_{i=1}^{I}\emptyset Q_{i}^{T}Q_{i}\emptyset^{T}X+\beta F_{U}^{H}y=\eta_{E\partial }+\beta F_{U}^{H}y, \end{array}$$

where $E_{\partial }=\sum_{i=1}^{I}\varphi Q_{i}^{T}P^{T}\left(\bar{x_{i}}\right)\emptyset \partial_{i}$,∑_*i*=1_^*I*^*Q*_*i*_^*T*^*Q*_*i*_=∧ is the diagonal matrix. The element on the diagonal corresponds to the position of the pixel in the image, and the value of the element represents the number of pixel overlaps. Because all pixels overlap the same number, there is

(12) $$\begin{array}{c} \sum_{i=1}^{I}\varphi Q_{i}^{T}Q_{i}\emptyset^{T}=pL. \end{array}$$

The reconstruction results of MRI image coefficients are as follows.

(13) $$\begin{array}{c} X={\left(\mu pL+\beta L\right)}^{-1}\left(\mu E_{\partial }+F_{U}^{H}y\right). \end{array}$$

The specific calculation process is as follows.

- Input initial image *y*, geometric direction *x*={*x*_1_, *x*_2_,…, *x*_*c*_,…, *x*_*C*_}, determination of *p*, regularization parameter *β*=10^8^, internal loop error limit *η*=5 × 10^−3^, and initial variable *X*=*F*_*U*_^*H*^*y*, *X*_last_=*X*, *η*=2^6^, *∂*_*i*_=0.
- When *η* ≤ 2^6^, determine *X*, calculating all *∂*_*i*_ and updating $E_{\partial }=\sum_{i=1}^{I}\varphi Q_{i}^{T}P^{T}\left(\bar{x_{i}}\right)\emptyset \partial_{i}$ at the same time.
- According to equation (13), *X*=(*μpL*+*βL*)^−1^(*μE*_*∂*_+*F*_*U*_^*H*^*y*)
- When ‖Δ*X*‖=*X*_last_ − *X* > *η*, *X*_last_=*X*, return to step b, and conversely, the next step is taken.
- *η* ≤ 2^6^, $\bar{X}\leftarrow X$, *μ* ← 2*μ*, return to step b
- Conversely, the algorithm terminates and the results are outputted

#### 2.3.3. Evaluation Indicators

The evaluation indexes of MRI and the image processing effect are commonly used as follows. When O and P are set to represent the width and height of the image, respectively, A, $\bar{A}$ represent the original image and reconstructed image, respectively.

(a) The equation for calculating signal noise ratio (SNR) is as follows.
  (14) $$\begin{array}{c} \text{SNR}=101\text{g}\left[\frac{255\times 255\times O\times P}{\sum_{a=1}^{O}\sum_{i=1}^{H}{\left(A\left(a,i\right)-\bar{A}\left(a,i\right)\right)}^{2}}\right]. \end{array}$$
(b) The calculation equation of relative *l*_2_ norm error (RLNE) is as follows.
  (15) $$\begin{array}{c} \text{PLNE}=\frac{{\left\|A-\bar{A}\right\|}_{2}}{{\left\|A\right\|}_{2}}. \end{array}$$
(c) The calculation equation of matching degree *γ* is as follows.
  (16) $$\begin{array}{c} \gamma =\frac{{\left\|\bar{A}\right\|}_{2-}{\left\|A\right\|}_{2}}{{\left\|\bar{A}\right\|}_{2+}{\left\|A\right\|}_{2}}. \end{array}$$

### 2.4. Immunohistochemical Detection

First, 3 mL venous blood was extracted on an empty stomach and centrifuged at a rotational speed of 3,000r/min for 10 min. After stratification, the supernatant was taken and stored at −70°C in a refrigerator for low temperature. Then, the serum malondialdehyde (MDA) level was detected by the colorimetric method, and the serum superoxide dismutase (SOD) was detected by the xanthine oxidase method. The instructions of the kit were strictly followed.

B cell lymphoma-2 (Bcl-2), Bcl-2-associated *X* (Bax), and Caspase-3 protein were detected by immunohistochemistry. The specific procedures are shown in Figure 2.

**Step 1 .**

The thickness of the section was paid attention to keep at 3 *μ*m.

**Step 2 .**

After the above dewaxing, hydration, repair, deionization, and other operations, the section was incubated in room temperature water for 15 min and repeatedly rinsed with buffer 3 times.

**Step 3 .**

After the operation of the step, it needs to be washed with buffer 1 time.

**Step 4 .**

Within the 8 hours of incubation, the temperature should be maintained at 4°C.

**Step 5 .**

After sheep anti-mouse IgM secondary antibody was addition-dropped biotin-labeled, it should be incubated for 20 min at room temperature before the subsequent operation.

### 2.5. Observation Indicators

MRI results of the two groups were compared before and on day 10 of treatment, including limb ischemia and blood perfusion. The levels of SOD and MDA in serum of the two groups were compared before and on the 10th day of treatment. The protein levels of Bcl-2, Bax, and Caspase-3 in two groups were compared before and on day10 after treatment.

### 2.6. Statistical Analysis

SPSS 22.0 statistical software was used for statistical analysis. The measurement data were expressed in ($\bar{x}$ ±*s*), the *t*-test was used, and the counting data were used the *χ*^2^ test. *P* < 0.05, the difference was statistically significant.

## 3. Results

### 3.1. Processing Effect of the Compression Reconstruction Algorithm Based on GPBDCT

Figure 3 shows the results of SNR, RLNE, and *γ* for the image processing effect evaluation indexes based on the GPBDCT-compression reconstruction algorithm and conventional compression reconstruction algorithm. SNR (22.01), RLNE (0.0792), and *γ* (0.9997) were better than the conventional compression reconstruction algorithm (*P* < 0.05). The image processing effect is shown in Figure 4. The image definition of Figure 4(c) is better than Figure 4(b).

### 3.2. Comparison of General Data

The gender distribution of the two groups was as follows: 70 males (51.85%) and 30 females (53.85%) in the observation group. There were 65 males (48.15%) and 35 females (46.15%) in the control group. Through calculation and analysis, there was no significant difference in the proportion of men and women between the two groups (*P* > 0.05), as shown in Figure 5. The average ages of patients in the two groups were as follows: (36.98 ± 5.78) years in the observation group and (37.50 ± 6.11) years in the control group. There was no significant difference in the comparison (*P* > 0.05), as shown in Figure 6. The mean values of S-S and ST in the two groups were as follows: (3.12 ± 0.61) h and (2.21 ± 0.18) h in the observation group and those were (3.21 ± 0.64) h and (2.39 ± 0.14) h in the control group. The comparison was not statistically significant (*P* > 0.05), as shown in Figure 7. The above results suggested the feasibility of comparison between the two groups.

### 3.3. MRI Results before and after Treatment

The MRI examination results of the two groups before treatment and on the 10th day of treatment were compared.  Figure 8 shows the MRI examination results of the observation group before and after treatment. Figures 8(a), 8(b), and 8(c) show the MRI examination results before treatment, and obvious high signal bleeding points could be observed. Figures 8(d), 8(e), and 8(f) show the MRI examination results on the 10th day of treatment, and the bleeding points were significantly reduced or even disappeared.  Figure 9 shows the MRI examination results of the observation group before and after treatment. Figures 9(a), 9(b), and 9(c) show the MRI examination results before treatment, and obvious high signal bleeding points could be observed. Figures 9(d), 9(e), and 9(f) show the MRI examination results on the 10th day of treatment, and the bleeding points were reduced, but there were still residues.

### 3.4. Serum SOD and MDA Levels

Table 2 shows the test results of SOD and MDA levels of the two groups before and after treatment. There is no significant difference between the two groups before treatment (*P* > 0.05). After treatment, the level of SOD (95.89 ± 11.21) U/mL in the observation group was significantly higher than that in the control group (81.37 ± 11.56) U/mL. MDA level (3.02 ± 1.78) *μ*mol/L was lower than that in the control group, (4.51 ± 1.98) *μ*mol/L, and the comparison was statistically significant (*P* < 0.05). Through calculation and analysis, the change degree of SOD and MDA levels between the two groups was compared. The change degree of SOD and MDA levels in the observation group was better than that in the control group (*P* < 0.05), as shown in Figure 10.

### 3.5. Bcl-2, Bax, and Caspase-3 Protein Levels

Table 3 shows the levels of Bcl-2, Bax, and Caspase-3 protein in the two groups before treatment. There was no significant difference in the levels of Bcl-2 (17.21 ± 3.02), Bax (11.01 ± 0.52), and Caspase-3 protein (377.32 ± 5.89) between the observation group and the control group before treatment (*P* > 0.05). After treatment, the expression of Bcl-2 protein in the observation group was higher than that in the control group, the expression of Bax and Caspase-3 protein was lower than that in the control group, and the difference was statistically significant (*P* < 0.05). Through calculation and analysis, the changes in Bcl-2, Bax, and Caspase-3 protein levels between the two groups were compared, and it was concluded that the changes in Bcl-2, Bax, and Caspase-3 protein levels in the observation group were better than those in the control group (*P* < 0.05) (Figure 11).

## 4. Discussion

Studies suggested that limb ischemia-reperfusion is closely related to diseases such as replantation of severed limbs, osteofascial compartment syndrome, and vascular injury of limbs [13]. Edaravone can treat ischemia-reperfusion diseases by scavenging free radicals [14]. In order to study the efficacy of edaravone in the treatment of lower limb ischemia-reperfusion injury, the MRI image processed by the CS image reconstruction algorithm based on curvelet transform of image block was employed to evaluate its efficacy.

The processing effect of the CS image reconstruction algorithm based on image block curvelet transform on MRI images was analyzed. It is concluded that the SNR (22.01), RLNE (0.0792), and *γ* (0.9997) of GPBDCT-based compression reconstruction algorithm are better than those of the conventional compression reconstruction algorithm. It is suggested that the optimization effect of this improved algorithm is better than that of the conventional CS reconstruction algorithm. Some research experts have also used the CS reconstruction algorithm improved by GPBDCT, SIDCT, and PBDCT algorithms for MRI image processing. The results show that the algorithm GPBDCT is better than SIDCT and PBDCT [15]. Dai et al. [16] conducted a similar study, suggesting that the ultrasonic block CS imaging reconstruction algorithm based on wavelet sparse representation can greatly reduce the total amount of data required for imaging and the number of data channels required for linear array transducers to receive data. Compared with the spatial frequency domain sparse algorithm, the imaging effect has been greatly improved. Then, the patients were rolled into two groups and treated them with edaravone and Mailuoning injections, respectively, analyzed, and compared the efficacy of the two treatment methods. According to the MRI results before and after treatment, the tissue bleeding caused by ischemia-reperfusion injury in the two groups has improved, but the observation group is significantly better than the control group.

A large number of studies have shown that edaravone can directly scavenge hydroxyl radicals through electrons and inhibit the chain reaction of cell membrane peroxidation, thereby effectively reducing the damage of intracellular oxygen free radicals [5, 17], to indirectly alleviate the bleeding caused by vascular endothelial cell injury. This study also analyzed the two groups of patients before and after treatment of serum SOD, MDA levels, and Bcl-2, Bax, and Caspase-3 protein levels. SOD can indirectly reflect the body's ability to scavenge oxygen free radicals, MDA belongs to an oxygen free radical, Bax is a proapoptotic gene, Caspase-3 is a multiple apoptotic pathway related factor, and Bcl-2 is mainly distributed in the mitochondrial membrane, and it not only can maintain the normal function of mitochondria and inhibit the spillover of apoptotic factors but also inhibit the release of calcium ions, playing a good role in antioxidant [18–20]. According to the above, the higher the levels of SOD and Bcl-2 are, the lower the levels of MDA, Bax, and Caspase-3 proteins are, indicating that the free radicals scavenging is better. This is consistent with the results of this study, and the therapeutic effect of the observation group is better than that of the control group. The changes in the levels of SOD (15 ± 2.02), MDA (2.27 ± 1.02), Bcl-2 (8.5 ± 1.02), Bax (3.7 ± 0.42), and Caspase-3 protein (35.9 ± 5.42) before and after treatment in the observation group are significantly higher than those in the control group, suggesting that edaravone has good treatment. Some studies have suggested that edaravone can significantly enhance the vitality of the IR flap and protect the flap blood vessels [21]. This is consistent with MRI findings.

## 5. Conclusion

MRI images based on the GPBDCT-compression reconstruction algorithm combined with other examination methods were adopted to evaluate the therapeutic effect of edaravone on lower limb ischemia-reperfusion injury. The results show that the GPBDCT-compression reconstruction algorithm has a better effect on MRI images, and edaravone can better remove free radicals and alleviate apoptosis. These results suggest that edaravone has a better therapeutic effect on lower limb ischemia-reperfusion injury after replantation of severed limbs and provides a more effective treatment for clinical patients. Due to the lack of research on the evaluation of related therapeutic effects by MRI, the research results lack certain comparison and authenticity. However, in this study, the results showed that edaravone had a good application prospect in the treatment of ischemia-reperfusion injury by scavenging free radicals.

## Figures and Tables

**Figure 1:** Image block results.

**Figure 2:** Detection steps of immunohistochemistry.

**Figure 3:** Comparison of evaluation results. (a) RLNE. (b) SNR. (c) *γ*. ^*∗*^Compared with routine, *P* < 0.05.

**Figure 4:** Treatment effect. (a) Original drawing. (b) Convention. (c) GPBDCT.

**Figure 5:** Distribution of men and women. (a) Men. (b) Women.

**Figure 6:** Average age comparison.

**Figure 7:** Comparison of S-S and ST.

**Figure 8:** MRI results of the observation group. (a), (d) Coronal plane. (b), (e) Transverse plane. (c), (f) Sagittal plane.

**Figure 9:** MRI results of the control group. (a), (d) Coronal plane. (b), (e) Transverse plane. (c), (f) Sagittal plane.

**Figure 10:** Changes of SOD and MDA levels in two groups before and after treatment. ^*∗*^Compared with the control group, *P* < 0.05.

**Figure 11:** Changes of serum Bcl-2, Bax, and Caspase-3 protein in two groups before and after treatment. ^*∗*^Compared with the control group, *P* < 0.05.

**Table 1:** MRI scan parameters.

Scan sequence	T1WI	T2WI	DEC-MRI	
			T1-vibe	T1-twist
TE (ms)	9	90	2	3
TR (ms)	205	3400	6	6
FOV (mm)	120 × 120	65 × 65	80 × 80	100 × 100
Layer thickness (mm)	3	3	3	3
Spacing (mm)	1	1	1	1
Matrix	256 × 256	120 × 120	130 × 130	130 × 130
Flip angle (°)	70	120	5/15	12
Layer number	9	9	9	9

**Table 2:** Statistics of serum SOD and MDA levels in the two groups.

Group	Observation group		Control group	
	Before treatment	After treatment	Before treatment	After treatment
SOD (U/mL)	80.89 ± 11.78	95.89 ± 11.21^*∗*^	81.37 ± 11.56	90.27 ± 10.42
MDA (*μ*mol/L)	5.29 ± 1.22	3.02 ± 1.78^*∗*^	5.38 ± 1.23	4.51 ± 1.98

*Note.* ^*∗*^Compared with the control group, *P* < 0.05.

**Table 3:** Serum Bcl-2, Bax, and Caspase-3 protein levels in two groups.

Group	Observation group		Control group	
	Before treatment	After treatment	Before treatment	After treatment
Bcl-2	17.21 ± 3.02	25.81 ± 4.01	18.01 ± 3.46	20.27 ± 3.42^*∗*^
Bax	11.01 ± 0.52	7.31 ± 0.28	10.79 ± 0.43	8.61 ± 0.43^*∗*^
Caspase-3	377.32 ± 5.89	341.42 ± 5.19	369.87 ± 5.21	358.78 ± 5.59^*∗*^

*Note.* ^*∗*^Compared with the control group, *P* < 0.05.

## Data Availability

The data used to support the findings of this study are available from the corresponding author upon request.
